# The N6-Methyladenosine- (m6A-) Associated Genes Act as Strong Key Biomarkers for the Prognosis of Pancreatic Adenocarcinoma

This article has been retracted.

**DOI:** 10.1155/2021/8715823

**Published:** 2021-11-19

**Authors:** Fei Li, Ping Zhang

**Affiliations:** Department of Pharmacy, Medical Supplies Center of PLA General Hospital, Chinese PLA General Hospital, Beijing 100853, China

## Abstract

**Background:**

Pancreatic adenocarcinoma (PAAD) has become the major cause of cancer-related deaths globally. The m6A (N6-methyladenosine) alteration plays a crucial function in carcinogenesis and tumor progression. The role of genes related to m6A and their expression level in pancreatic cancer is not identified yet. The objective of this research analysis is a demonstration of the m6A RNA methylation regulators based as biomarkers for the PAAD diagnosis.

**Methods:**

About 23 extensively reported m6A RNA methylation regulators were identified through the Cancer Genome Atlas (TCGA) database. This identification was based on consensus clustering analysis, protein-protein integration (PPI) analysis, risk prognostic model, Cox-regression analysis, String Spearman analysis, and LASSO Cox-regression.

**Results:**

Herein, we conclude that 23 m6A methylation regulators have a strong link with the clinical and molecular characteristics of PAAD. The three subgroups (1/2) of pancreatic adenocarcinoma were identified using the clustering of 23 m6A regulators. Subgroup cluster 2 had a lower survival rate than the subgroup of cluster 1, and the difference in grades between the two groups was substantial. An assessment was performed using the 23 reported m6A methylation regulators. Eight of these can be used as independent PAAD prognostic markers. The consequences of variable IGF2BP3 expression in PAAD were then investigated further.

**Conclusions:**

The key finding of this study was that the m6A methylation regulator gene has the main role in pancreatic tumors, and it may be used as a biomarker in the prognosis of the PAAD and for therapy purposes.

## 1. Background

PAAD is one of the commonly occurring malignant tumors in the digestive system in the world. According to the American Cancer Society, in 2019, 23,800 deaths for men and 21,950 deaths for women occurred due to PAAD in the United States [1]. By 2030, in malignant tumors, PAAD became the second major cause of mortality. [2]. Tumor genetic studies have found that PAAD has many recurrent genetic changes, including the deletion of TP53, SMAD4, and CDKN2A, as well as activation of KRAS [3]. Currently, surgery is the only treatment for PAAD. Although, there is not only a need for sustainability of PAAD patients [4]. However, the prognosis has improved slightly recently, the survival rate for 5 years after disorder is still below 5% [5]. Therefore, finding new treatment methods and prognostic markers for PAAD is crucial.

In the 1970s, geneticists explored that m6A is present in mRNA [6]. Many methylation modifications occur on mRNAs such as N6-2-O-dimethyladenosine (m6A-m) and N7-methyloguanosine (m7G) but m6A is a potential modification that occurs in eukaryotic mRNAs. As a representative in the epitranscriptome, m6A mRNA modifications participate in many vital activities in the cell such as differentiation of the stem cells, self-renewal, mRNA transcription, nuclear export, alternative splicing, translation (protein synthesis), micro-RNA (miRNA) processing, and degradation. These processes determine the expression or inactivation of specific genes, which is vital for growth and development. M6a reader (YTHDC1) helps promote exon-inclusion with the help of certain arginine and serine splicing factors. [7]. Reduced METTL3 or WTAP in zebrafish governs various abnormalities in development and progressive metastasis [8]. m6A could dynamically alter the secondary structure of mRNA and regulate mRNA-protein interactions affecting the alternative splicing of mRNA [9]. m6A expression level is significantly increased by the low level (knockdown) of YTHDF-2 and it is also used to inhibit the prostate cancer cell migration and proliferation. Further tests revealed that miR-493-3p and YTHDF2 were correlated harmfully and that miR-493-3p targets YTHDF2's 3′UTR directly. MiR-493-3p forced expression dependably raises m6A levels while inhibiting tumor expansion and progression. [10].

Recent studies revealed that m6A alteration has a crucial role in various types of illnesses (including hypertension, cardiovascular disease, and malignancies) [11–13]. It has also been revealed that detection of the m6A-genes and m6A-RNA methylation regulators functions for the prognosis of different tumors as biomarkers. Multiple investigations have discovered the functionality and regulation of m6A in different kinds of tumors. m6A affects the expansion, differentiation, invasion, and progression of various tumors. The m6A methyltransferase complex, for example, is mostly made up of methyltransferase-like 3 (METTL3), METTL14, METTL16, and Wilms' tumor 1-associating protein (WTAP), all of which work together to control m6A distribution. The main component is METTL3, whereas METTL14 is a stable heterodimer that catalyzes m6A RNA methylation through a correlative impact with METTL3 [14]. Because WTAP lacks a methyltransferase mechanism, this balancing component operates on the assumption that the m6A methylation complex is functioning [15]. METTL16, a recently identified m6A writer that targets U6 spliceosomal short nuclear RNA, also controls S-adenosylmethionine balance by increasing S-adenosylmethionine synthetase production in response to methionine deficiency. [16]. Previous studies had no comprehensive or systematic approach to diagnosis of cancer because they had considered only one or two m6A-genes/m6A RNA methylation regulators.

In the following research, we hypothesized that m6A is a new prognostic marker and new drug target for PAAD. We conducted a detailed analysis of 23 commonly reported genes linked to m6A RNA methylation. For this purpose, we used the TCGA database for RNA seq data.

## 2. Materials and Methods

### 2.1. Data Retrieval

The UCSC Xena (http://xena.ucsc.edu/) and Genotype-Tissue Expression (http://commonfund.nih.gov/GTEx/) both databases were applied to retrieve the transcriptome data of PAAD patients that are linked with TCGA datasets. This data has purely relied on clinical data, e.g., gender, age, stage, grade, and TNM stage survival status including survival time. UCSC Xema contains the RNA seq transcriptomic data and respective physiological characteristics of PAAD patients. On the other hand, GITEX is used to collect RNA-transcriptome data from human healthy tissues [17]. A total of 185 tumor samples from eight data set samples have valid prognostic information, which can be used to construct and evaluate predictive models. The TCGA datasets' clinicopathological parameters are summarized (Additional file 1).

### 2.2. Screening of m6A RNA (de)Methylation Genes

Genes related to m6A-methylation were selected from previous studies [18, 19]. Using the Limma program, deferentially expressed genes (DEGs) were screened between diseased samples (PADD samples) and control samples. For the selection of DEGs, the cutoff threshold values were set at adjusted P0.05 and absolute log2FC > 1 [20]. A gene expression matrix of 23 genes was extracted. The extracted data was utilized in the bioinformatics analysis that followed.

### 2.3. Correlation and Consensus Cluster Analysis

The STRING database (version 11.0, http://string-db.org) was applied to perform the protein-protein interaction analysis among the m6A regulators [21]. The research species was defined as “human.” The lowest interaction score was set to 0.900; from this interaction score, all disconnected nodes in the network are hidden. The rest of the parameters were kept the same as the default settings. For identification of network connections among the m6A-methylation regulators, the Pearson correlation model was applied. To check the m6A methylation regulators and their expression levels, whether it is related to prognosis or not, the TCGA PAAD cohort was distributed into different dissimilar groups using the ConsensusClusterplus in R, relied on coexpression of m6A-methylation regulators [22]. The difference in overall survival among various clusters was analyzed by utilizing the Kaplan Meier and log-rank tests. Chi-square assessment was applied for dispersal analysis of the gender, age, stage, grade, N.T stage, and survival status among various clusters.

### 2.4. Prognostic Signature Generation and Prediction

Evaluation of the association between the m6A regulators (m6A-RNA methylation regulators) and OS in TCGA PAAD cohort was done using survival analysis in R based on the univariate cox regression model. Genes with risk ratios (HRs) greater than one are considered dangerous, while genes with an HR lower than one are considered protective. The prognostic signatures of eight genes were determined (KIAA1429, also known as VIRMA, METTL16, IGF2BP3, HNRNPC, RBM15, PCIF1, METTL3, YTHDF1, IGF2BP2, and ALKBH5). The best model was found using multivariate Cox regression analysis. Then, using an L1-penalized (LASSO) method, the chosen genes with independent prognostic significance were further identified [23]. Finally, the minimal requirements were used to estimate their regression coefficients. The given equation was used to calculate the risk score of the signature.

(1) $$\begin{array}{c} \text{Risk}\_\text{score}=\sum i=1n\text{Coefi}*xi, \end{array}$$

In the above equation, “Coefi” is the coefficient of regression, and “xi” indicates the expression level of every analyzed gene. According to this formula, the risk score of each patient was evaluated by the multiplication of each gene expression with its coefficient. The TCGA PAAD had two main groups including low risk and high risk, dependent on the average risk score. Two tests such as Kaplan Meier and log-rank were applied to compute the distinguishing features in OS between the high risk and low risk groups. The construction receiver-operating characteristic curves (ROC) were used to assess the precision of the prognostic model's prediction [24]. A chi-square test was used to evaluate the clinicopathological characteristics' distribution between the low-risk group and high-risk group of genes. The differences between heatmap R packages were shown using heatmaps. The independent prognostic variables based on the TCGA PAAD cohort were determined using single-factor and multifactor Cox regression models. The distinguishing features of survival duration between low- and high-risk groups of genes were investigated depending on the gender, age, stage, grade, T.N stage, and survival status.

### 2.5. Bioinformatics Analysis of m6A Methylation Genes Related to Prognosis

cBioportal (http://www.cbioportal.org/index.do) web-server [25] provided useful information for the PAAD patients having m6A-genes' mutations. The target connectivity relationship of the m6A-methylation genes and miRNA was identified using the miRWalk-database (mirwalk.umm.uni-heidelberg.de) [26]. The therapeutic characteristics and related genes of IGF2BP3 in PAAD and normal samples, as well as other tumor subgroups, were analyzed and queried using UALCAN database (working under the cBioportal for the cancer omics data) [27]. Gene ontology and pathway enrichment analysis were used to find the association of the IGF2BP with PADD.

### 2.6. Statistical Analysis

One-way variance based on gender, survival time, age, stage, survival status, T, N stage, and grade was applied to evaluate the difference in expression levels of 23 regulator genes in normal tissues and diseased tissues. This analysis was performed on 179 diseased samples (PAAD patients) and 171 control samples from pancreatic tissues of the TCGA datasets. Before the construction of the scoring model, a tool survminer was applied to evaluate the optimum cutoff for each risk score in the training group. After finding the optimal cutoff value, cells were divided into low- and high-risk groups regarding the optimum cutoff value. ROC curve was applied to assess the risk scoring model's prediction accuracy (AUC). ANOVA and co-ANOVA regression models were used to investigate the different cancer diagnostic factors such as gender (male vs. female), age (60 vs. >60), risk score, and PAAD subtype. For all statistical analysis R versions, 3.6.0 was utilized, and a significant *P* value was confined as less than 0.05.

## 3. Results

### 3.1. The Expression Level of the Genes Related to m6A Differs among Tumor and Control Samples

The genes related to m6A methylation are shown in Table 1. Expression patterns of genes related to m6A regulators among the diseased (PAAD) and controlled samples were analyzed with the help of heatmaps (Figure 1(a)) generated by R. In tumor samples, ALKBH5, YTHDF3, ZC3H13, YTHDF2, RBM15, PCIF1, YTHDF1, IGF2BP1, IGF2BP3, and IGF2BP2 were notably superior in normal control samples, while METTL14, ALKBH3, METTL16, YTHDC2, YTHDC1, HNRNPA2B1, HNRNPC, METTL3, RBMX, WTAP, KIAA1429, and FTO were significantly reduced in the tumor samples. The values of the gene expression differences are shown in Figure 1(b).

### 3.2. Interactions and Connections of Methylation Regulators of m6A-RNA

Figure 2(a) shows interaction among 23 methylation regulators of m6A RNA. HNRNPA2B1 and HNRNPC might be central genes of the interaction network. The related analysis further supported the verification results of the interactive network. Furthermore, the interaction between HNRNPA2B1 and HNRNPC m6A RNA methylation regulators, both HNPNPC and METTL3 and YTHDC1 and METTL3 had a high positive correlation (*r* = 0.89). HNRNPC was adversely linked with YTHDF1 (*r* = 0.89), and METTL3 was negatively correlated with YTHDF1 (Figure 2(b)).

### 3.3. Three Clusters with Clinical Outcomes Related to Pancreatic Adenocarcinoma Were Identified by the Clustering of Methylation Regulators of the m6A-RNA

PAAD patients' population can be separated into three subgroups of clusters such as cluster 1; cluster2 (*K* = 2) relied on the similar expression of the methylated regulators of the m6A-RNA; this is shown in Figures 3(a)–3(c). Clinical characteristics of the two groups (normal samples and diseased samples) were shown in Additional file 2. Preclassification by clustering process was employed on the samples and two clustering groups were made. In the 1st group, 79 samples were positioned and named that cluster as cluster 1, and in the 2^nd^ group, 99 samples were placed and named that cluster as cluster 2. Principal component analysis was used to find the transcriptional patterns' difference between the cluster-1 and cluster-2.

The findings revealed substantial differences and their existence between these two groupings (Figure 3(d)). A significant reduction of OS was assessed in cluster-2 compared to cluster-1 (*P* = 3.396 × 10^−04^). This analysis was done using the Kaplan Meier program. Reduction of OS indicated that 23 methylation regulators may have a critical role at the prognostic level (Figure 3(e)). From the current study, it was revealed that group 1 has a greater survival rate of 476 days, but group 2 has less survival rate of 393 days. This study also focused on the relationship of clinicopathological properties and clustering that revealed that there were greater deviations between the survival status and grading about *P* = 0.05 but no significant variations were observed in T, N, and stage (Figure 3(f)).

### 3.4. Documentation of Prognostic Signature

The methylation regulators of m6A-RNA linked with the overall survival (OS) and PAAD cohort were identified by univariate coregression analysis. Results showed that these regulators such as METTLL16 (*P* < 0.001), HNRPC (*P* = 0.032), KIAA-1429 (*P* = 0.008), IGF2BP3 (*P* < 0.001), METTL-3 (*P* = 0.023), RBM-15 (*P* = 0.013), YTHDF-1 (*P* = 0.013), PCIF1 (*P* = 0.007), ALKBH-5 (*P* < 0.001), and IGF2BP2 (*P* < 0.001) were highly linked with the OS in TCGA PAAD cohort. KIAA-1429, IGF2BP3, IGF2BP2, HNRNPC, and RBM-5 have safeguarded genes with an HR less than 1, while METTL16, PCIF1, METTL3, YTHDF1, and ALKBH5 are hazardous genes with an HR more than 1. (Figure 4(a)). The LASSO technique was used to calculate coefficients for these 10 genes, which were used to create prognostic markers. One hundred and seventy-six PAAD patients were divided into two clusters such as high-risk group and low-risk group. The survival rate of the higher and lower risk groups was different in PAAD patients; patients in the higher risk group showed low survival rates, but on the other hand, patients in the lower risk group showed a high survival rate (*P* = 5.011*e* − 04) (Figure 4(b)). The distribution of two risk scores based on gene signatures is shown in Figure 4(c).  Figure 4(d) represented the distribution analysis of the risk scores and overall survival status (OS-status). The AUC value of the prognostic-prediction model was 0.803. This value was the indication of the high prediction efficiency of the signature model shown in Figure 4(e). METTL16, PCIF1, METTL3, and YTHDF1 have high expression in the low-level risk, while KIAA1429, IGF2BP2, IGF2BP3, and HNRNPC have high expression in the high-risk group (Figure 4(f)). A remarkable difference existed in grade (*P* 0.05) and survival status (*P* 0.01) between the low-risk and high-risk groups.

### 3.5. TCGA PAAD Cohort, the Risk Score Based on Diagnosis Signatures Is an Independent Diagnostic Factor

To test if the risk score based on diagnostic indicators is an independent diagnostic predictor, researchers used ANOVA and co-ANOVA Cox regression analysis. Following the deletion of instances with missing *M* values, 175 cases were used for further investigation. Age (*P* = 0.016, HR = 1.028, 95 percent CI = 1.0051.051), N (*P* = 0.003, HR = 2.258, 95 percent CI = 1.3083.898), and risk score (*P* 0.001, HR = 17.969, 95 percent CI = 7.09545.510) were all significantly associated with OS in ANOVA analysis (Figure 5(a)). When these variables were investigated through the multivariate Cox proportional hazard regression, the same behavior in risk score was found (Figure 5(b)). In the TCGA PAAD dataset, the results showed that age and risk score were self-determining prognostic variables. The gene signature generated from the 8 m6A-associated genes was shown to have independent prognostic significance and good prediction accuracy, according to our findings.

### 3.6. Mutations and miRNA Prediction Analysis of m6A-Associated Genes

To study the potential mechanism of action of the m6A-associated genes in PAAD, the genetic mutation analysis shown in Figures 6(a) and 6(b) reveals that the mutation percentages of HNRNPC, IGF2BP2, IGF2BP3, KIAA1429, METTL3, METTL16, PCIF1, and YTHDF1 were 1.8%, 2.4%, 1.2%, 5%, 1.2%, 0, 0.6%, and 1.8%, respectively. In the miRWalk database, we used the mirTarBase database as the screening threshold. There were 18 miRNAs targeting HNRNPC, four miRNAs targeting IGF2BP2, and four miRNAs targeting YTHDF1. There were four miRNAs targeting IGF2BP3, two miRNAs targeting METTL16, and one miRNA targeting VIRMA (Figure 6(c)). Those are useful for clarifying the molecular mechanism of m6A-associated genes in PAAD.

### 3.7. Investigation of IGF2BP3 Expression in PAAD

The mRNA binding protein 3 or insulin-like growth factor II (IMP3 or IGF2BP3) is part of the insulin-like growth factor II or mRNA binding proteins family. IGF2BP3 was originally identified in pancreatic cancer [28], and it has since been revealed to be strongly identified in many cancer tissues, including colon cancer, hepatic cancer, lung cancer, and cervical cancer [29]. IGF2BP3's elevated expression in cancer tissues might point to its involvement as an oncogene in carcinogenesis. The further study discovered that IGF2BP3 is the translation activator of IGF IImRNA, which relies on IGF II to drive the proliferation of leukemia cells [30]. IGF2BP3 is now thought to be a particular tumor biomarker in colorectal cancer as research progresses [31].

Further subgroup analysis of various clinical-pathological features of 179 PAAD samples in TCGA has consistently shown high transcription levels of IGF2BP3. According to a subgroup analysis of gender, drinking habits, diabetes status, pancreatitis, nodal metastasis status, and TP53 mutation, the transcription level of IGF2BP3 in PAAD patients had a higher percentage as compared to healthy people (Figures 7(a)–7(f)). The enrichment analysis of GO and KEGG with positively related genes found that the genes by their positive correlation are intimately connected to the biological behavior of tumors and can directly regulate the signaling pathway of PAAD (Figures 7(g) and 7(h), Additional file 3). Therefore, IGF2BP3 performs functions in the progress of PAAD and may become a clinical prognostic indicator.

## 4. Discussion

The onset and progression of PAAD are varied phase phenomenon involving the gradual acquisition of genetic and epigenetic changes, resulting in the uncontrolled growth and proliferation of tumor cells. Therefore, it is crucial to clarify the potential molecular events that cause PAAD tumors. It has also been revealed that abnormal modifications of m6A methylation are involved in activating several types of tumors [32].

The regulation by ALKBH5 is reduced in chronic pancreatitis, resulting in increased m6A levels and decreased regulation by the tumor suppressor gene KCNK15-AS1, allowing pancreatic tumor cells to migrate and invade more easily [33]. Some recent studies found that pancreatic cancer is caused by the overexpression of the YTHDF2 that is involved in two cellular processes such as epithelial-mesenchymal transition (EMT) inhibition and proliferation [34].

Studies revealed that METTL3 is overexpressed in prostate cancer, and it controls the Hedgehog pathway. It was discovered that the hedgehog pathway promotes prostate tumor growth by bringing alterations in m6A and by promoting the expression of GLI zinc finger-1 (GLI-1) which is a crucial part of the Hedgehog pathway [35]. Furthermore, METTL3 was shown to be substantially elevated in hepatoblastoma and to accelerate its progression [36].

Their function in PAAD, however, is unknown. Herein, we identified 23 genes and their role in regulating the m6A-RNA methylation mechanism. Our study also revealed that these 23 genes are expressed abnormally in PAAD disease. Furthermore, two subgroups of TCGA PAAD were made on the dependent coexpression of the m6-A-related genes having substantial variations in tumor grade and survival status. More crucially, the signatures of these eight genes were effectively validated as independent prognostic markers in the external independent PAAD cohort, showing that the model for the prognosis had a higher rate of accuracy and efficiency in the prognostic prediction process.

Previous studies have been shown that methylation genes related to m6A are expressed improperly in different types of cancers; they have no consistent expression level. In ovarian cancer, for example, YTHDF1 is frequently increased; it is also observed that overexpression of the YTHDF1 is not suitable for the cancer prognosis. It is directly linked with a poor prognosis. The multiomics studies on ovarian cancer identified that EIF3C acts as a direct target for the YTHDF1. YTHDF1 increases the incidence and spread of ovarian cancer by increasing the EIF3C m6A-dependant mechanism of translation, and this is accomplished by the binding of the YTHDF1 with the modified EIF3C m6A-mRNA [37]. Our findings show that ten of the 23 m6A RNA methylation regulators in PAAD samples were upregulated, while twelve were downregulated, suggesting that these genes may be related to cancer cell carcinogenicity and/or PAAD patient prognosis. To figure out what's going on at the molecular level, further study is needed.

There were two clustering groups related to PAAD identified using consensus clustering. The identified groups were recognized dependent on regulations of the m6A-genes. A major distinction was observed in survival status and tumor grading among the two clustering groups suggesting that m6A-regulators' expression is directly linked with PAAD's poor prognosis. One of the study's key results was the identification of eight genetic risk factors, including IGF2BP3 and METTL3, as well as the evidence that multiple independent cohorts can accurately predict PAAD patients' prognosis. The main difference is observed in overall survival (OS) among low- and high-risk groups after dividing the clinicopathological features into two PAAD cohorts. It was also observed that the clinical features of high risk-group were not favorable than the low-risk group.

The m6A-regulators may have opposing roles in the same or different kinds of cancers.

In endometrial cancer and glioblastoma, for example, METTL3 operates as a tumor suppressor gene [38], but as an oncogene in gastric cancer [39]. Our prognostic model indicates that IGF2BP3 expression is adversely associated with PAAD prognosis, indicating that IGF2BP3 is a PAAD oncogene. Applying the Gene Ontology (GO) and pathway (KEGG) analysis of the positively linked genes with IGF2BP3, it was found that these genes are involved in pancreatic cancer pathways, p53 signaling pathways, cell cycle processes, pathways that are significantly related to tumorigenesis and its development, and cell to cell connections. It further describes the important role of IGF2BP3 in pancreatic cancer and is likely to become a new diagnostic and screening biomarker for pancreatic cancer. Recently, fewer researchers have done about the role of IGF2BP3 in the development of PAAD. Taniuchi et al. reported that IGF2BP3 promotes invasion and metastasis of PAAD through a local translation of IGF2BP3-binding transcripts. This indicates that IGF2BP3 may play a part in the carcinogenesis of PAAD [40]. The expression level of the IGF2BP3 was significantly enhanced in ovarian clear cell carcinoma. The experimented studies exhibited to be contrasted with the control group; the tumor size was considerably reduced after treatment with IGF2BP3siRNA. This also shows that IGF2BP3 has a cancer-promoting effect in OCCC [41]. In addition, the incidence of PAAD is closely related to changes in people's eating habits, smoking, heavy drinking, acute and chronic pancreatitis, type 2 diabetes, and stimulation by exposure to physical and chemical substances. Diabetic patient has the more chances of pancreatic cancer due to the direct link with the pancreas [42]. Our study also revealed that the chances of PAAD in patients with old diagnosis diabetes were increased by 52%, and the PAAD risk in patients with newly onset diagnosed diabetes (duration less than 3 years) was increased 2.3 times higher than the old, diagnosed patients with diabetes. Naudin et al. found that drinking was positively correlated with the risk of PAAD in men, but not significantly correlated with the risk of PAAD in women. Their study also found that beer and spirits have a higher carcinogenic risk than wine [43]. Acute pancreas cancer is among the risk factors for PAAD. Kirkegard et al. found that the chances of incidence of PAAD in patients with acute pancreatic cancer have been increased almost eight times after five years of diagnosis [44]. Inflammatory reactions can damage DNA and lead to abnormal DNA damage repair. Chronic inflammation is a long-term process. Long-term and continuous stimulation of body cells leads to the accumulation of damage, which greatly increases the risk of tumors. Our study also found that IGF2BP3 showed significant differences in diabetes, chronic pancreatitis, alcohol consumption, and gender compared with normal controls. It is assumed that IGF2BP3 may also promote PAAD through the above pathogenic factors.

In order to detect the content and location of RNA modifications, researchers have developed a variety of quantitative or fixed-point RNA modification detection methods using liquid chromatography, mass spectrometry, and high-throughput sequencing. These methods are convenient and economical and have good feasibility. Presently, molecular techniques such as high-performance liquid chromatography (HPLC), 2D cellulose thin layer chromatography (2DTLC), liquid chromatography, and coupling of liquid chromatography with mass spectrometry (LCMS) are used for the RNA quantification. RNA site-specific detection technology has gradually developed from the low-throughput primer extension technology and SCARLET technology in the past to the commonly used high-throughput sequencing technology [45]. These technologies, therefore, provide strong support for the feasibility of clinical testing of m6A-biomarkers for the prognosis of PAAD patients.

## 5. Conclusion

This research focused on the expression, protein-protein interactions, possible function, and PAAD prognostic significance and genes for methylation related to m6A-RNA. The expression of m6A genes in PAAD is linked to malignant clinicopathological characteristics, according to our findings. This indicates that the prognostic marker aids as a reliable molecular marker to monitor the development of PAAD and provides a significant guiding strategy for the selection of treatment methods and the development of new drugs.

## Figures and Tables

**Figure 1:** The expression levels of m6A RNA methylation regulators in the TCGA PAAD cohort. A heatmap was utilized for visualization of the regulation levels of m6A RNA methylation regulators in all cancer samples. (b) Deferentially expressed methylated regulators of m6A were shown in normal and cancer samples, green color represented normal samples, and orange represented tumor samples. ^∗^*P* < 0.05, ^∗∗^*P* < 0.01, and ^∗∗∗^*P* < 0.001.

**Figure 2:** Protein-protein interaction network (PPI) and correlative examination of the regulators of the m6A-related genes. (a) showed the interaction network among the m6A-regulators. (b) showed the correlation analysis of m6A-gene-related regulators using the Pearson correlation model. In this figure, crosses mean there was no correlation.

**Figure 3:** Overall survival analysis and three differential characteristics of pancreatic adenocarcinoma (PADD). (a) showed the cumulative distribution function (CDF) in which *K* = 2‐9. (b) showed that the area is changed relatively under the “CDF curve” in which *K* = 2‐9. (c) represented the matrix (*K* = 2) for the consensus clustering. (d) showed the mRNA expression profile using PCA in TCGA dataset (principal component analysis) analysis; patients with PAAD disease were placed in cluster 1 represented by red color, and the patients in cluster 2 represented in green. (e) showed the overall survival (OS) for clusters 1 and 2 using the Kaplan Meier curves. (f) represented by heatmaps showing the clinicopathological characteristics of the two subgroup clusters (1 and 2).

**Figure 4:** Prognostic signature was constructed using the TCGA PAAD cohort. (a) Identification of correlated genes with OS by the univariate regression analysis of the methylation-regulated genes of m6A-RNA. (b, c) are used to show the computed coefficients by the Cox regression analysis. (d) explained that the overall survival rate was less in the high-risk group of clustering than the low clustering risk group. (e) is used to represent the evaluation of the prediction efficacy of the prognostic model. (f) was showing a high difference rate for the fastest and grade between the low-risk group and the high-risk group.

**Figure 5:** This figure was utilized to represent the self-regulating variables and identification from the TCGA PAAD cohort. (a) explained that correlated indicators with OS were demonstrated by applying the univariate regression analysis and clinicopathological features of risk score. (b) Independent prognostic factors were identified by applying the multivariate analysis and clinicopathological characteristics of the risk score.

**Figure 6:** Genomic alterations and miRNA-target regulatory network of m6A-related prognostic genes involved in human tumors, demonstrated by cBioportal and miRWalk database analysis of TCGA databases. (a, b) Alteration frequency of m6A-related prognostic genes in PAAD patients. (c) Predicted miRNA-target by miRWalk3.0.

**Figure 7:** IGF2BP3 transcription in subgroups of PAAD. (a) Relative expression level of the IGF2BP3 in normal individuals and PAAD patients either in male or female was shown using the box plot. (b) Relative expression of IGF2BP3 in PAAD patients or normal individuals with drinking habits was shown using the box plot. (c) In this figure, relative expression was shown in PAAD patients or normal persons at diabetes status. (d) was showing the relative expression of the IGF2BP3 in normal or PAAD patients at pancreatic status. This expression was shown by a box plot. (e) was used to explain the expression level of IGF2BP3 in normal or PAAD patients for the nodal metastasis; box plot was used for this purpose. (f) In this figure, box plot was applied to show the relative expression level of IGF2BP3 in regular or PAAD patients with TP53 mutations. (g) showed the Gene Ontology investigation of the positively related genes with IGF2BP3. (h) showed the analytical mechanism of the highly correlated genes with IGF2BP3. The mean of data was ± SE. ^∗^*P* < 0.05; ^∗∗^*P* < 0.01; ^∗∗∗^*P* < 0.001.

**Table 1:** m6A methylation-related genes.

Official symbol	Function
METTL3	Catalyzes m6A modification
METTL14	Balances the assembly of MTC and demonstrates detailed RNA sequence
METTL16	Catalyzes m6A modification
YTHDC1	Promotes RNA splicing and export
YTHDC2	Improves the protein synthetic activation of target mRNA while reduces the profusion of target mRNA
YTHDF1	Promotes mRNA translation
YTHDF2	Promotes mRNA degradation
YTHDF3	Interacts with YTHDF1 to promote mRNA translation/interacts with YTHDF2 to promote mRNA degradation
WTAP	Recruits METTL3 and METTL14 into the nuclear speckles
VIRMA	Recruits the MTC and correlates with polyadenylation cleavage factors, CPSF6 and CPSF5.
FTO	Removes m6A modification
HNRNPA2B1	Promotes primary miRNA processing
HNRNPC	Regulates mRNA abundance and splicing
RBMX	Regulates mRNA abundance and splicing
ZC3H13	Combines with WTAP to keep MTC in the nuclear speckles
ALKBH3	Removes m6A modification
ALKBH5	Removes m6A modification
EIF3A	Induces mRNA recruitment to the 43S PIC and detects the mRNA for AUG recognition.
IGF2BP1/2/3	Enhances the constancy and protein synthesis from mRNA
PCIF1	Recruits to the early elongation complex of RNAPII via interaction with POLR2A and mediates the formation of m6A(m) cotranscriptionally

## Data Availability

All the studied and analyzed data are present in this research article.

## Abbreviations

METTL3: Methyltransferase-3
METTL14: Methyltransferase-14
METTL16: Methyltransferase-16
YTHDC1: YTH domain comprising 1
YTHDC2: YTH domain comprising of 2
YTHDF1: YTH N6-methyladenosine RNA-binding protein 1
YTHDF 2: YTH N6-methyladenosine RNA-binding protein 2
YTHDF3: YTH N6-methyladenosine RNA-binding protein 3
WTAP: WT1-associated protein
VIRMA: vir-like m6A methyltransferase-linked
FTO: FTO alpha-ketoglutarate dependent dioxygenase
HNRNPA2B1: Heterogeneous nuclear ribonucleoprotein A2/B1
HNRNPC: Heterogeneous nuclear ribonucleoprotein C
ZC3H13: Zinc finger CCCH-type containing 13
ALKBH3: alkB homolog 3, alpha-ketoglutarate-dependent dioxygenase
ALKBH5: alkB homolog 5, RNA demethylase
IGF2BP1: Insulin-like growth factor 2 mRNA-binding protein 1
IGF2BP2: Insulin-like growth factor 2 mRNA-binding protein 2
IGF2BP3: Insulin-like growth factor 2 mRNA-binding protein 3
PCIF1: PDX1 C-terminal inhibiting factor 1
RBMX: RNA-binding motif protein X-linked
CI: Confidence interval
EIF3A: Eukaryotic translation initiation factor 3 subunit A
PAAD: Pancreatic adenocarcinoma
HR: Hazard ratio
ROC: Receiver-operating characteristic
AUC: Area under the curve
TCGA: The Cancer Genome Atlas
OS: Overall survival.
